# A Pulmonary Artery-Vein Separation Algorithm Based on the Relationship between Subtrees Information

**DOI:** 10.1155/2021/5550379

**Published:** 2021-06-09

**Authors:** Kun Yu, Ziming Zhang, Xiaoshuo Li, Pan Liu, Qinghua Zhou, Wenjun Tan

**Affiliations:** ^1^Key Laboratory of Intelligent Computing in Medical Image, Ministry of Education, Shenyang 110189, China; ^2^College of Medicine and Biological Information Engineering, Northeastern University, Shenyang 110189, China; ^3^College of Computer Science and Engineering, Northeastern University, Shenyang 110189, China

## Abstract

Physicians need to distinguish between pulmonary arteries and veins when diagnosing diseases such as chronic obstructive pulmonary disease (COPD) and lung tumors. However, manual differentiation is difficult due to various factors such as equipment and body structure. Unlike previous geometric methods of manually selecting the points of seeds and using neural networks for separation, this paper proposes a combined algorithm for pulmonary artery-vein separation based on subtree relationship by implementing a completely new idea and combining global and local information, anatomical knowledge, and two-dimensional region growing method. The algorithm completes the reconstruction of the whole vascular structure and the separation of adhesion points from the tree-like structure characteristics of blood vessels, after which the automatic classification of arteries and veins is achieved by using anatomical knowledge, and the whole process is free from human intervention. After comparing all the experimental results with the gold standard, we obtained an average separation accuracy of 85%, which achieved effective separation. Meanwhile, the time range could be controlled between 40 s and 50 s, indicating that the algorithm has good stability.

## 1. Introduction

Pulmonary artery-vein (A/V) separation of CT images is important to fit downstream medical tasks quantitatively in clinic. In CT images, pulmonary arteries and veins overlap in many places. The discrimination of arterial from venous irrigation is challenge because of (1) the limited scanning resolution of CT image, (2) the relatively high spatial density of pulmonary blood vessels, and (3) the part of the volume and size effect. These factors also lead to complexity in separating arteries and veins in pulmonary CT images [1]. Meanwhile, the classification of arteries and veins is also of great practical significance for diagnosis of chronic obstructive pulmonary diseases (COPDs) and the detection of lung tumors, which attracts many efforts to the development of this area [2]. The separated arteries and veins can be more visually presented to the physician, allowing for more accurate and effective patient care, as well as providing a wealth of information for the development of vascular surgery strategies.

At the beginning, some geometric and artificial methods were proposed, but they have great limitations. Nakamura et al. [3] have proposed a pulmonary vascular classification method based on the spatial arrangement of blood vessels using the distance of the bronchus from the blood vessels and the distance of interlobar fissures from the closest pulmonary blood vessels. However, there are only three cases included in the study, which limited its generality. A tracking-based automated method for low-dose CT scans to separate arteries from other surrounding structures has been introduced by Wala et al. [4]. The algorithm starts from automatically detected seed points located in the basal pulmonary areas and continues by tracking the vessel and detecting bifurcations. A quantitative evaluation of results reported 64% sensitivity and 90% specificity values. Using multiscale opening operators, Saha et al. [5] have also separated the arteries and veins of different sizes and locations based on two sets of manually selected seeding points. The disadvantage of the above two methods lies in the manual collection of seed points, which requires a high degree of professionalism and increases the workload of doctors. Gao et al. [6] then have improved Saha's semiautomatic method by embedding a 2D-3D interconnected graphical user interface to achieve 91%–95% accuracy, but they still have the effort consuming problem caused by user intervention. The method used by Park et al. [2] is to construct minimum spanning trees and cut edges to separate arteries and veins. Although it can effectively achieve the separation, manual optimization is still needed.

Later automatic separation methods were proposed, and neural networks were used for A/V separation. Kitamura et al. [7] proposed an automatic A/V separation method. It uses energy minimization of high-order potentials and selects higher-order clusters based on prior knowledge of data and the desired shape. This method has been evaluated in 10 sets of CT data. However, only the pulmonary vessels with CT values greater than 200 HU have been considered, which to certain extent impairs its universality. A classification method based on a deep learning novel and powerful method for dealing with non-Euclidean data is presented, while Convolutional Neural Network (CNN) framework has been proposed recently [8]. Using a 3D CNN method, small blood vessels are extracted directly from noncontrast CT images to learn specific A/V characteristics without further operation. However, the model is only evaluated for its ability to diagnose COPD in the article, which lacks a validated evaluation of the accuracy for A/V separation. More recently, a new framework to approach the separation of tree-like structures using local information along with a specifically designed graph-cut methodology has been proposed [9]. It employs a random forest (RF) preclassifier to exploit the local anatomical differences of arteries and veins. The experiments reveal a relevant improvement in the accuracy of the vessel classification with the proposed framework compared to using only local information. Graph Convolutional Networks (GCNs) are a powerful method for dealing with non-Euclidean data, while CNNs can learn features from Euclidean data such as images [10]. In Zhai et al.'s work, they propose a novel method to combine CNNs with GCNs (CNN-GCN), which can consider both Euclidean and non-Euclidean features, to separate the pulmonary vascular trees into arteries and veins (A/V) [10]. It shows a better performance compared with CNN method but slightly worse results compared to observers, which needs a further improvement.

Here, we propose a novel algorithm for pulmonary artery-vein (A/V) separation. In this method, local and global information, anatomic knowledge, and 2D area growth method are involved, aiming to solve the above-mentioned problems in pulmonary arteries and veins separation. An average accuracy of 85% has been achieved in the overall process. The processing time is ranging between 40 s and 50 s, indicating good performance and stability of this algorithm. Our new method may provide a new idea for the A/V classification of CT images.

## 2. Materials and Methods

### 2.1. Geometric Graph Representation and Separation

The pulmonary vasculature can be abstracted as a feature tree with a certain logical structure maintaining the original vascular topology. Such trees can be bifurcated structures, trinomial structures, and so on. The classification of vessels essentially separates the adhesion points on the CT map so that the arteries and veins form two separate trees.

Due to the morphological complexity, pulmonary blood vessels appear to be bifurcations, trifurcations, artery-vein attachments, and false positives in CT images, making it difficult for a centerline algorithm to deal with them. On the other hand, the centerline algorithm shows good structural characteristics when the vessels are locally disturbed by noise or false positives [11]. Therefore, this paper starts with centerline algorithm, employing a geometric graph representation to roughly separate vascular branch structures and nonvascular structures.

Ideally, a normal bifurcated vessel will be a pixel connected with three adjacent pixels (Figure 1(a)). The relevant information about a center point (a node) and its 26 neighbors can be stored in a data structure as follows: idx represents the location information of the pixels based on which adhesion point is calculated (some are more than one); links represent the index matrix of a link to which the adhesion point is connected; conn represents the index matrix of a node adjacent to the adhesion point;com_*x*, com_*y*, com_*z* represent the *x*, y, and *z* coordinates of the adhesion point, respectively; and ep is equal to either 0 or 1, where 0 represents the nonleaf nodes and 1 represents the leaf nodes. The connectivity is defined within the 26 neighbors, and edges represent a voxel collection of two adjacent points, shown as a simple tubular structure.

A link structure includes 3 parts as follows: *n*_start represents the index value of the starting pixel; *n*_end represents the index value of the end pixel;points represent the index value of all pixels contained in the link. Each node and link can represent any morphological structure mentioned above, i.e., bifurcations, trifurcations, attachments, end points, or false positive structures. Once a data structure of a node is known, we can obtain its neighborhood topology through the link property information. As shown in Figure 1(b), we can easily identify tri- and multifurcation through this transformation. The corresponding nodes are shown as yellow circles. The rest of the circles are leaf nodes colored blue. Branches are divided into red and black colors, where black represents branches connected to the leaf nodes, and the rest are colored red.

When a length of a link (the value of the property “links”) is greater than 3, there will be four or more blood vessels connected around the certain node. This node is then regarded as an adhesion point of arteries and veins. After detecting the adhesion points, an originally continuous link will be split into two links. Take quadfurcations as an example, the coordinates of the central adhesion point are set to (*x*, *y*, *z*), and the coordinates of the two leaf nodes with an unknown angle are set to A (*x*_1_, *y*_1_, *z*_1_) and B (*x*_2_, *y*_2_, *z*_2_), respectively. The rearrangement of four links will be done by calculating the angles (*θ*) between branches with a single leaf node and their adhesion point, according to the following equations:

(1) $$\begin{array}{c} a_{1}={\left(x_{1}-x\right)}^{2}+{\left(y_{1}-y\right)}^{2}+{\left(z_{1}-z\right)}^{2}, \end{array}$$

(2) $$\begin{array}{c} b_{1}={\left(x_{2}-x\right)}^{2}+{\left(y_{2}-y\right)}^{2}+{\left(z_{2}-z\right)}^{2}, \end{array}$$

(3) $$\begin{array}{c} c_{1}={\left(x_{1}-x_{2}\right)}^{2}+{\left(y_{1}-y_{2}\right)}^{2}+{\left(z_{1}-z_{2}\right)}^{2}, \end{array}$$

(4) $$\begin{array}{c} \text{pos}=\frac{\left(a_{1}+b_{1}-c_{1}\right)}{\left(2*\text{sqrt}\left(a_{1}\right)*\text{sqrt}\left(b_{1}\right)\right)}, \end{array}$$

(5) $$\begin{array}{c} \theta =\arccos\left(\text{pos}\right)*\frac{180}{\pi }. \end{array}$$

According to the above quadfurcation, there will be three different combinations. The combination with the maximum value of *θ* will be adopted. Meanwhile, a new pair of links will be regenerated to represent the original four links. Both the intrinsic property of the original adhesion node and the connected links are then modified. For different links passing through adhesion points, a separation is made to ensure they belong to a different class.

### 2.2. Combination of Subtrees

Starting with the leaf nodes, connected links are classified into many different classes. In practice, the sub_trees can only belong to either an arterial class or a venous class. The reduction of links classification is achieved by a flowchart shown in Figure 2. Starting with the leaf nodes, connected links can be classified into the same class. After this operation, the adhesion points in a subtree can be removed, leaving only zero and trifurcations. Pulmonary blood vessels have been divided into a set of subtrees based on local information.

### 2.3. Relationships between Subtrees

In the next steps, we will extract the relationship between the subtrees using global information. Peripheral matching is applied to establish the relationship between subtrees. This method is based on anatomic knowledge that (1) arteries and veins meet at alveolar sacs and (2) arteries and veins are approaching each other rather than connected to each other [11, 12]. Thus, a one-to-one relationship can then be built based on the spatial location of the leaf nodes from two subtrees without knowing the classes. By analyzing each leaf node of a subtree and finding the closest leaf node from another subtree within a Euclidean distance, peripheral matching defines the matching strength between two subtrees (IMS) increasing by 1. A higher IMS indicates two subtrees likely belonging to different classes of blood vessels. To reduce the coincidence of establishing this relationship, a minimum value of IMS between the two vascular subtrees is required (Figure 3).

Peripheral matching can describe the relationship between two subtrees with the value of IMS. However, in some cases, it is still unknown whether there is a relationship between two subtrees if they do not have an IMS value. For this situation, we can establish indirect class relationships through the known relationships. For example, for three subtrees *S* = {*ψ*_1_^*A*^, *ψ*_2_^*B*^, *ψ*_3_^*C*^}, the exact A/V classes information of A, B, and C is unknown. However, both subtrees of class A and C, and class B and C have a high IMS. It is easy to infer that A and B belong to a different class compared to C. Since there are only two classes, subtree A and subtree B then belong to the same class of subtrees. After the division of relationships between subtree classes, the number of different subtree types in the geometric graph can be further reduced.

### 2.4. Restoration of Vascular Tree

Before distinguishing the specific class of blood vessels, a restoration of vascular tree based on geometric graph is conducted. Each pixel point is used as a seed point for a two-dimensional (2D) region growing. A new dataset is constructed and the corresponding vascular subtree is exported until all data slides are processed. Through this restoration procedure, an intact tubular structure of pulmonary blood vessels can be built (Figure 4), which will facilitate the further classification step.

### 2.5. Classification of Blood Vessels

The final task is to classify these vascular trees by the volume differences between arteries and veins. Based on anatomical knowledge, the overall volume of venous trees is higher than arterial trees. Thus, the total volume of subtrees belonging to the same class is extracted from the vascular segmentation. A volume of each class per unit length is used, where the class with the highest volume is classified as veins and the other class as arteries. At this stage, the majority of subtrees have been classified. However, for subtrees with only a few leaf nodes, there is not enough peripheral information to establish a matching relationship. This kind of subtrees cannot connect to any others. To ensure the continuity of vascular labeling, each leaf node needs to connect to the root node through just one path. At each node in this path, the next direction is given by maximizing the branch angle and minimizing the difference in the diameter of the blood vessels between the front and back edges. For some unlabeled subtrees, there may be more than one path to the root node. They are classified by a majority vote of the already classified edges. If there are more subtrees in these paths that belong to the veins, then the unlabeled subtree belongs to the venous class; otherwise, it belongs to the arterial class.

## 3. Results and Discussion

To evaluate the performance of our method, 10 sets of CT image data from a top first-class hospital are used. The data resolution is 512 × 512, and the number of data layers is between 368 and 436. In order to verify the accuracy of pulmonary A/V separation, the data of the extracted topology of pulmonary blood vessels are used for experiments. All experiments are conducted using MATLAB 2015b and Visual Studio 2010 on a PC with Intel® Core™ i5-6700 CPU @ 3.40 GHz processor, 8.00 GB memory, and 1 TB Western Data hard drive.

As shown in Figure 5, each set of data is converted into geometric graph representations (Figures 5(e)–5(h)) from centerlines (Figures 5(a)–5(d)). Examples of details from corresponding geometric graphs are shown in Figures 5(i)–5(l), where both nodes and branches are divided into two categories. Leaf nodes are represented in blue color, adhesion nodes are colored yellow, branches connected to leaf nodes are colored black, and the rest of the branches are colored red. This representation will facilitate the acquisition of topological relationships between nodes and branches. For the nodes at the adhesion points with more than 3 branches, a geometric graph separation process is carried out. These adhesion points are taken as central points, and the branches belonging to the same blood vessel are connected together. A successful separation and reassembly of the adhesion points have been achieved based on the spatial structure of the blood vessel branches.

A depth-first traversal method is then employed to link different subtrees. A collection of subtrees are reconstructed based on the previous results, each of which is a subtree containing only bifurcations and trifurcations. The subtrees are further combined into the same class based on their relationships. The obtained two types of subtrees are marked with red and blue, respectively (Figures 5(m)–5(p)). An artery-vein classification is finally achieved based on 2D region growing method. As shown in Figure 6, pulmonary arteries are colored red, and pulmonary veins are colored blue.

We next evaluate the experimental performance. During the whole process, some adhesion points with five or more branches are not fully separated due to their structural complexity, which results in a misjudgment of the A/V separation. Here, a preliminary accuracy rate is obtained from the ratio of misjudged branches to the total number of the branches. The accuracy of the separation of the right and left lungs was similar at about 85% at different levels. However, as the number of layers increased, the accuracy of both left and right lung separation decreased slightly and the running time increased slightly.

Moreover, the final separation accuracy is obtained by comparing the experimental results with the gold standard with an average accuracy of 85% (Table 1). The processing time of the whole process/algorithm is then recorded. The running time of all five experiments described above exhibits a smooth line within the time range between 40 s and 50 s (Table 1), indicating a good stability of this algorithm.

## 4. Conclusions

This work achieves an automatic A/V separation by a method combining both global and local information. Firstly, a geometric graph is built based on the centerlines; next, a separation of the adhesion points is performed by applying the information of the geometric graphs; subtrees are then combined according to the local and global information; the combined subtrees are growing into vascular trees by using 2D area growth method; and finally the arterial and venous vascular trees are classified based on the knowledge of anatomy. The average accuracy of the overall process can reach 85% which is promising for a clinical application.

Currently, there are relatively few studies that perform automatic arteriovenous separation with both global and local information. This study can serve as a guide in the treatment of lung diseases such as pulmonary nodules and lung tumors. In future studies, we will investigate how we can differentiate arterioles more quickly and accurately.

## Figures and Tables

**Figure 1:** Schematic diagram of centerline to geometry: (a) centerlines of blood vessels; (b) geometric graph representation.

**Figure 2:** Flowchart of reducing subtree classification.

**Figure 3:** Flowchart of the peripheral matching of the subtree.

**Figure 4:** Schematic diagram of the vascular subtrees.

**Figure 5:** Schematic diagram of the pulmonary vascular geometric graph representation: (a–d) centerlines reconstructed based on Dataset 1 (a, b) and Dataset 2 (c, d), among which a and c are right lungs, and b and d are left lungs; (e–h) horizontally corresponding geometric graph representation; (i–l) graphic details of corresponding representations; (m–p) subtree separation results.

**Figure 6:** Schematic diagram of pulmonary arteriovenous vascular tree: (a) Dataset 1, right lung; (b) Dataset 1, left lung; (c) Dataset 2, right lung; (d) Dataset 2, left lung.

**Table 1:** Accuracy of pulmonary arteriovenous separation.

Dataset	No. of layers	Statistic of branches				Separation accuracy (%)		Running time (s)
		Total number of branches in the left lung	The number of misjudged branches in the left lung	Total number of branches in the right lung	The number of misjudged branches in the right lung	Acc of left lung (%)	Acc of right lung (%)	
1	368	943	123	532	59	86.76	85.74	46
2	386	498	68	506	70	86.34	86.03	49
3	378	624	84	587	85	85.74	85.12	52
4	403	486	79	619	95	83.79	84.64	48
5	436	536	89	472	74	83.40	84.32	52
Average						85.20	85.17	49.4

## Data Availability

The data used to support the findings of this study are available from the corresponding author upon request.
